The article "Involvement of Nucleotide Excision and Mismatch Repair Mechanisms in Double Strand Break Repair" was published in 2009. Journal: Curr Genomics.

# Involvement of Nucleotide Excision and Mismatch Repair Mechanisms in Double Strand Break Repair

**DOI:** 10.2174/138920209788488544

**Published:** 2009-06

**Authors:** Ye Zhang, Larry H Rohde, Honglu Wu

**Affiliations:** 1 NASA Johnson Space Center, Houston, Texas 77058; 2 University of Houston at Clear Lake, Houston, Texas 77058, USA

**Keywords:** Ionizing radiation (IR), DNA damage, DSB repair, NER, MMR and cell cycle.

## Abstract

Living organisms are constantly threatened by environmental DNA-damaging agents, including UV and ionizing radiation (IR). Repair of various forms of DNA damage caused by IR is normally thought to follow lesion-specific repair pathways with distinct enzymatic machinery. DNA double strand break is one of the most serious kinds of damage induced by IR, which is repaired through double strand break (DSB) repair mechanisms, including homologous recombination (HR) and non-homologous end joining (NHEJ). However, recent studies have presented increasing evidence that various DNA repair pathways are not separated, but well interlinked. It has been suggested that non-DSB repair mechanisms, such as Nucleotide Excision Repair (NER), Mismatch Repair (MMR) and cell cycle regulation, are highly involved in DSB repairs. These findings revealed previously unrecognized roles of various non-DSB repair genes and indicated that a successful DSB repair requires both DSB repair mechanisms and non-DSB repair systems. One of our recent studies found that suppressed expression of non-DSB repair genes, such as XPA, RPA and MLH1, influenced the yield of IR induced micronuclei formation and/or chromosome aberrations, suggesting that these genes are highly involved in DSB repair and DSB-related cell cycle arrest, which reveals new roles for these gene products in the DNA repair network. In this review, we summarize current progress on the function of non-DSB repair-related proteins, especially those that participate in NER and MMR pathways, and their influence on DSB repair. In addition, we present our developing view that the DSB repair mechanisms are more complex and are regulated by not only the well known HR/NHEJ pathways, but also a systematically coordinated cellular network.

## INTRODUCTION

Environmental DNA-damaging agents, including ultraviolet (UV) and ionizing radiation (IR), are constant threats causing DNA damage in living organisms. There are different forms of DNA damage, including double-strand break (DSB), as well as other types of damages such as hydrolytic depurination, apyrimidinic sites, and oxidative damage to the bases and the phosphodiester backbone of DNA. Repairs of different types of DNA damage are believed to follow lesion-specific repair pathways, such as DSB repair, nucleotide excision repair (NER), mismatch repair (MMR), or base excision repair (BER) [1]. Specific groups of proteins from these pathways recognize DNA damage sites, and repair and induce cell cycle checkpoints. After sensing a genotoxic agent-induced primary DNA damage, a series of signal transduction cascades are initiated that are responsible for arresting the damaged cells at the cell cycle checkpoints, maintaining cellular homeostasis, and sending signals to interact with neighboring cells. For example, early responses to DNA damage caused by IR are the activations of protein kinases ATM/ATR (ataxia telangiectasia mutated/ Rad3-related) and the downstream p53 signaling pathway [2-4]. Subsequently, transcriptional regulation of various genes and post-translational modification of proteins involved in DNA damage sensing, repair, and cell cycle regulation occur so that additional cascades of signaling pathways are initiated [5, 6].

The article "Involvement of Nucleotide Excision and Mismatch Repair Mechanisms in Double Strand Break Repair" was published in 2009. Journal: Curr Genomics.

Among all types of DNA damage, DSB is the most serious form that affects both strands of the DNA duplex. DSB is the major DNA damage induced by IR, including gamma and X- rays, although it does cause other minor damage to DNA [7]. Some chemotherapy drugs, such as bleomycin, mitoxantrone, amsacrine and etoposide, induce DSBs as well [8-10]. DSBs make cells more prone to unsuccessful DNA repair due to the lack of a complementary template, especially in G1 phase cells. Unrepaired DNA damage may cause cell cycle arrest and apoptosis; however, the accumulation of misrepairs may lead to chromosome instability and carcinogenesis. The two distinct pathways for DSB repair that have been identified are homologous recombination (HR) and non-homologous end joining (NHEJ), serving in two different scenarios [11-13]. DSB repair through HR requires the homologous sister chromatid or homologous chromosome, which only appears in late S/G2 phase, resulting in the error free restoration of the missing information to the damaged DNA [12]. However, in G1/early S-phase, the NHEJ pathway may contribute the most to DSB repair. This can lead to an error prone repair due to its joining of the two ends of broken DNA without a homologous template [13]. The success of DNA repair through these two mechanisms requires the same Rad50-MRE11-NBS1 complex with two distinct groups of proteins, which have been studied for decades.

Damage to the DNA that does not produce a DSB is repaired by the BER, NER, or MMR pathways. NER is capable of recognizing and repairing a large variety of DNA helix-distorting lesions, including UV induced pyrimidine dimers and DNA intrastrand cross-links [14, 15]. Two distinct processes of NER, global genomic NER (GG-NER) and transcription coupled NER (TC-NER), are involved in damage repair of transcriptionally silenced or active areas of the genome, respectively. The mechanisms of these two pathways are similar except for damage recognition. MMR, which occurs mostly at the post-replication stage, is responsible for repairs of mismatches and small stranded DNA loops that are important in stabilizing the genome. The MMR mechanism is also believed to interact directly with NER and homologous recombination [16, 17]. Defects in these DNA repair mechanisms produce gene mutations, which are associated with several syndromes, such as xeroderma pigmentosum (XP), and can significantly increase the possibility of oncogenesis [18, 19]. Recent studies have presented increasing evidence that these non-DSB repair mechanisms are highly involved in DSB repair. These findings, which are the focus of this review, have dramatically widened the current knowledge of DSB repair mechanisms and have indicated that the various DNA repair pathways are not separated, but well interlinked.

The article "Involvement of Nucleotide Excision and Mismatch Repair Mechanisms in Double Strand Break Repair" was published in 2009. Journal: Curr Genomics.

## NER PROTEINS IN DSB REPAIR

More than 30 proteins are required in a successful NER process to finish a series of tasks including damage recognition, DNA duplex opening, damaged DNA strand cutting, DNA synthesis, and strand ligation. Helical distortion of the DNA duplex and modification of the DNA chemistry are the common features of lesions recognized by the NER pathway [20]. In GG-NER, the XPC protein complex is responsible for the initial detection of damaged DNA [21], whereas, in TC-NER, the displacement of a stalled RNA Polymerase complex is aided by the CSA and CSB proteins in order to allow the NER proteins to access the damaged site [22]. There is substantial evidence that suggests three NER complexes, namely XPC/HR23B, XPA/RPA and ERCC1/XPF, may actively be involved in DSB repair. Genes associated with the NER pathway, such as XPC, have been found to be consistently up-regulated by IR [23, 24]. It has been found that the XPC defect affects the expression of some DSB repair genes induced by cisplatin, which causes DNA cross-links [25]. Various reports have suggested that XPC defects elicit impaired cellular responses to IR, indicating the possible role of XPC in DSB repair. Recently, Biard and his research group reported that long-term suppression of the XPC gene in HeLa cells changed DNA repair capacity by affecting NHEJ DNA repair, although the expression of NHEJ proteins were not altered [26]. The deficiency of XPC resulted in 30-40% reduction of NHEJ efficiency with decreased intramolecular joined products, thus affecting the cellular response to acute high dose IR-induced DNA damage. XPC knock-down (XPC^KD^) cells also exhibited an enhanced sensitivity to etoposide (VP16), a topoisomerase II inhibitor that creates DSBs through the progression of DNA replication forks [26].Moreover, both XPC^KD^ and HR23B^KD^ HeLa cells displayed intolerance to high dose gamma rays, showing increased cell cycle arrest and decreased survival based on clonogenic assays [27]. Furthermore, an XPC deficient cell line derived from an XP-C patient also showed disrupted cellular response to gamma rays [28]. To date, more than a hundred polymorphic variants in the XPC gene have been identified. Among the three most common polymorphisms, Ala499Val (C-T), PAT (-/+) and Lys939Gln (A-C), Lys939Gln (A-C) has been reported to be associated with reduced DNA damage repair capacity in human peripheral blood leukocytes (PBLs) after gamma ray exposure [29, 30]. This may explain the increased risk of malignancies associated with this variant allele of XPC [31-33]. These results reveal that the XPC protein is involved in DSB repair and may act in a much broader cellular mechanism than initiation of GG-NER alone.

The article "Involvement of Nucleotide Excision and Mismatch Repair Mechanisms in Double Strand Break Repair" was published in 2009. Journal: Curr Genomics.

Although the initial recognition step is different between the GG- and TC-NER pathways, the subsequent step in both pathways is essentially identical with the binding of the XPA/RPA complex to the injury site that supports damage recognition and subsequent repair machinery recruitment [34, 35]. First identified as a single-strand DNA binding protein in the 1990s, heterotrimer RPA consists of 70 (RPA1), 34 (RPA2) and 14 kD subunits and is found to be involved in diverse DNA metabolic activities and the NER pathway to maintain genomic stability through both *in vivo* and *in vitro* approaches [36, 37]. Later studies have suggested that RPA plays a role in DSB repair and in almost every DNA repair mechanism. RPA participates in these processes through its interaction with other proteins and its strong affinity for single-stranded DNA (ssDNA) [37, 38]. Recombinant RPA was first found to have a physical interaction with RAD52 proteins *in vitro* and in insect cells [39]. RPA also colocalized with RAD51 to form foci in IR irradiated exponentially growing mouse fibroblasts [40]. Further studies have shown that the phosphorylated form of RPA2 has cellular interaction with RAD52, as well as ATR in response to genotoxic insults [41]. In various human cells receiving IR treatment, RPA2 has been found to relocate to form distinct nuclear foci, colocalized with gamma-H2AX at the sites of DNA damage in a time-dependent manner. This reaction was phosphatidylinositol-3 (PI-3) kinase and ATM dependent. The time course of RPA and gamma-H2AX foci formation correlated well with the DSB repair activity analyzed by neutral comet assay [42]. The depletion of RPA by small interfering RNA (siRNA) elevated the frequencies of IR-induced micronulcei (MN) and apoptosis [42].

The article "Involvement of Nucleotide Excision and Mismatch Repair Mechanisms in Double Strand Break Repair" was published in 2009. Journal: Curr Genomics.

Many studies have also been conducted on other species, such as *Saccharomyces cerevisiae (S. Cerevisiae)*, and find that RPA has a direct role in homologous recombination repair, which is essential for the repair of DNA DSBs in mitotic and meiotic cells. RPA directly binds to RAD52 upon replication stress and the depletion of the RPA protein inhibits the formation of RAD51 nuclear foci in the presence of persistent unrepaired DNA DSBs led by hydroxyurea-induced replication stalling [43]. After decades of various studies, Kowalczykowski’s group has proposed a mechanism of second-end capture as one of the DSB repair steps, which involves RPA as the initial protein binding to the 3’ ssDNA tails of the resected DSB [44, 45]. Another *in vitro* study showed that NHEJ proceeded faster and to higher levels of completion in the presence of recombinant RPA protein, although this DSB rejoining was apparently not RPA dependent. The results suggest that in addition to its role in homologous recombination, RPA may also have a supportive role in some forms of non-homologous end-joining [46]. In our earlier study, the loss of RPA1 expression impaired DSB repair, as shown by increased MN formation, indicating the important function of RPA during the process of DNA repair [47].

It is believed that XPA is involved in DNA damage recognition and also in the recruitment of other NER factors to the DNA damage site to form dual incision complexes through protein-protein interactions [48, 49]. It has been shown that XPA has high affinity to ds-ssDNA junctions and interstrand crosslink lesions (ICLs), the common DNA intermediate structures in many DNA metabolic pathways, suggesting the additional role of XPA beyond the NER pathway [50, 51]. In our former study, gamma irradiated cells with suppressed expression of XPA exhibited a phenotype of elevated cell cycle progression and higher incidence of MN, as well as a higher frequency of chromosome translocations, indicating involvement of XPA in the regulation of DSB repair [47]. This may explain why, in addition to XP syndrome, a higher incidence of spontaneous tumorigenesis has been observed in the *Xpa^-/-^* mice compared to wild type controls [52, 53].

In the next step of the NER process, the endonucleases XPG and ERCC1 (Excision Repair Cross-Complementing Group-1)/XPF are recruited to the damaged site and cleave one strand of the DNA at positions 3' and 5' to the damage, respectively. This step generates a displaced strand of about 30 oligonucleotides in order to proceed with the gap repair synthesis [54-56]. XPF has been shown to be physically involved in psoralen and mitomycin C induced ICL repair [57, 58], indicating that the ERCC1–XPF complex may have functions in cellular processes other than the NER pathway, such as DNA recombination and double-strand break repair. The homolog proteins of ERCC1-XPF in various species do facilitate DSB repair and mediate the resistance to IR [59-61]. Similar findings have provided substantial evidence that the ERCC1-XPF complex mediates DSB repair in both normal mammalian cells and mouse embryonic stem cells. ERCC1-XPF deficient murine and human fibroblast cells showed hypersensitivity to IR similar to cells defective in HR-mediated or NHEJ DSB repair [62]. Furthermore, the involvement of ERCC1-XPF may be Ku independent since ERCC1^-/-^ KU86^-/-^ fibroblasts were more sensitive to gamma irradiation compared to single mutants and Ercc1^-/- ^DNA-PKs^-/-^ double mutants, causing a significant persistence of gamma H2AX foci and accumulation of chromosomal aberrations. It suggests that ERCC1-XPF may be an alternative DNA end-rejoining factor, but not be a part of traditional NHEJ machinery because there is no evidence of severe NHEJ deficiency in *Ercc1^-/-^*, *Xpf^-/-^* mice or humans with XPF deficiency [63]. However, *Ercc1/Xpf* mutant mice did show hypersensitivity to gamma irradiation, establishing an essential role for ERCC1-XPF in protecting against DSBs *in vivo*. The XPF deficiency has been shown to be responsible for a pronounced genomic instability phenotype with suppressed gene conversions in the Chinese hamster cell line UV41 [63]. It suggests that single strand annealing (SSA) may be the alternative pathway for HR or NHEJ repair of DSBs, which is ERCC1-XPF dependent. SSA was first identified in *S. Cerevisiae *[64]. The DSB lying between two repeated sequences can stimulate the deletion between the repeats, annealing of these two complimentary sequences, and DNA synthesis and ligation through this SSA pathway [64, 65]. Many DSB repair proteins as well as several mismatch repair proteins, such as Rad52, RPA and MSH2, are involved in the SSA pathway [65-67]. A recent report from Helleday’s group has provided evidence that ERCC1-XPF may mediate the repair of DSBs through both SSA and gene conversion pathways in homologous recombination [68].

The article "Involvement of Nucleotide Excision and Mismatch Repair Mechanisms in Double Strand Break Repair" was published in 2009. Journal: Curr Genomics.

## MMR PROTEINS IN DSB REPAIR

The MMR system is responsible for the post-replicative repair of mismatches and small single-strand DNA loops. There are several proteins engaged in the MMR process, including two different heterodimeric complexes of MSH2-MSH3 and MSH2-MSH6 with different misrepair recognition specificity. Another heterodimeric complex of MLH1-PMS2 interacts with MSH complexes and replication factors. Excision and resynthesis of the misrepaired strand are performed by a number of proteins, such as PCNA and RPA. Most importantly, the MMR pathway is believed to serve as one of the most critical genome surveillance systems to maintain faithful DNA replication and transmission of accurate genetic information [69-71]. It has been suggested that MMR proteins are broadly involved in various aspects of DNA metabolism, such as the DNA damage response and homologous recombination which mediate DSB repair, rather than DNA mismatch correction alone. Defects in this system, such as mutations in MSH2 and MLH1, may be involved in the process of oncogenesis and have been reported to be associated with various cancers, including hereditary nonpolyposis colorectal cancer [72, 73].

In *S. Cerevisiae*, homologous recombination initiated by DSBs proceeds through two distinct pathways, gene conversion and SSA [74, 75]. In both cases, any presenting nonhomologous DNA at the ends must be removed before new DNA synthesis and ligation can occur and this event depends not only on the NER endonuclease RAD1/RAD10 but also on MSH2 and MSH3 [76-78]. Defects in MSH2 and MSH3 have been shown to impair the removal of nonhomologous ends in both DSB-induced gene conversion and SSA [79]. It has been confirmed that *S. cerevisiae* MSH2-MSH3 specifically binds branched DNA substrates containing 3' single-stranded DNA and the release of MSH2-MSH3 is ATP-dependent. This binding of MSH2-MSH3 to the double-strand/single-strand junction enables the change of DNA conformation to an open position [79]. Researchers further confirmed that MSH2-mutant embryonic stem (ES) cells fail to correct mismatched heteroduplex DNA (hDNA) that is formed adjacent to the DSB during gene conversion repair of DSBs although cells seemed to be able to repair DSBs efficiently. This suggests that gene conversion repair of DSBs in mammalian cells involves mismatch repair proteins [80]. Another study showed that MSH2-deficient colorectal carcinoma cell lines failed to accurately repair enzyme restricted plasmid DNA DSBs mediated by gene conversion [81]. Compared with more than 50% in MSH2-proficient cells, only 8% of MSH2 deficient cells presented precise gene conversion products, resulting in significant increase of rearranged repair [81]. Moreover, a recent study by Waldman’s research group has verified that MSH2 deficient CHO cells produce less precise gene conversion products, although the overall frequency of DSB-induced recombination was increased [82]. All these reports suggest that MSH2 modulates homologous recombination. In response to genotoxic insults, *Msh2*^-/-^ murine embryonic fibroblasts and *Msh2*-deficient mouse colorectal carcinoma cells were hypersensitive to CPT-induced chromosomal damage and cell death [83]. In the absence of MSH2, the recruitment of RAD51 to the damage sites is delayed [83]. X-ray irradiated MSH2-deficient cells showed the absence of MRE11 or RAD51 relocalization and reduced cell survival, which were associated with increased chromosomal damage in G2 phase cells [84]. In addition to altered HR associated with MSH2 deficiency, loss of MSH2 may also influence the NHEJ pathway at the step of pairing of terminal DNA tails [85]. These impaired responses of MSH2-deficient cells to genotoxic insults indicate the involvement of MSH2 in the repair of DSBs.

The article "Involvement of Nucleotide Excision and Mismatch Repair Mechanisms in Double Strand Break Repair" was published in 2009. Journal: Curr Genomics.

MLH1, another protein involved in MMR repair, has also been suggested to be involved in the DSB repair pathway and reported to be required in the NF-kappaB activation after treatment with both CPT and X rays [86]. Although *Mlh1^-/-^* mouse embryonic fibroblasts had similar NHEJ efficiency to that of control cells to repair an I-SceI restricted plasmid that is stably transfected into the cells, the incidences of deletion associated with NHEJ events were dramatically higher in wild-type cells. This indicates that MLH1 modulates error-prone NHEJ by inhibiting the annealing of DNA ends containing noncomplementary base pairs [87]. Furthermore, the influence of MLH1 on IR-induced autosomal mutations has been studied in a mouse *Mlh1^-/-^* kidney cell line. A high frequency of IR induced mutations was found in *Mlh1^-/-^* cells due to increased crossover events of mitotic recombination, suggesting that MLH1, or MMR may serve as a modulator in mitotic HR repair [88]. *Mlh1^-/-^* mice, which have been used as a model of hereditary non-polyposis colorectal cancer (HNPCC), spontaneously developed gastrointestinal tumors (GIT) and thymic lymphomas by 48 weeks. X-ray irradiation of *Mlh1 *knockout mice has been found to accelerate the carcinogenesis process of GIT [89]. Our data in a previous study showed that the expression of MLH1 was induced by IR, and the loss of MLH1 expression not only elevated cell cycle progression but also increased the yield of IR-induced chromosomal translocations, suggesting that this gene, involved mostly in MMR, may play a role in DSB repair and cell cycle regulation [47].

## NER AND MMR PROTEINS IN DNA DAMAGE-INDUCED G2-CELL CYCLE ARREST

The DNA double strand break repair and checkpoint control are the two major mechanisms that function to prevent chromosomal instability following exposure to DSB inducers, such as IR. ATM has been identified as a critical factor for the initiation of checkpoint pathways [90]. The substrates of ATM kinase are broad, including many cell cycle control proteins participating in G1/S and G2/M checkpoint pathways [2, 91-95]. It is still poorly understood how the initial DNA lesion signals the initiation of checkpoints, and how the successful DNA repair allows the release of cells through the checkpoints. Recent studies have suggested that DNA repair proteins may be involved in cell cycle signaling and act beyond their repair roles. DNA damage repair processing by repair proteins may be required for recruiting checkpoint proteins to damaged DNA to activate checkpoints. MMR and NER have both been shown to not only regulate DSB repair, but also to be involved in IR induced cell cycle arrest, especially the G2/M checkpoint. In diploid growth cells, two different proposed G2/M arrest mechanisms may be present in mammalian cells [96]. The G2/M checkpoint that occurs early and transiently after IR is ATM dependent, and prevents cells in G2 phase at the time of irradiation from progressing into mitosis. The next stage is G2/M accumulation, which is measurable several hours after IR. This later event of G2/M arrest is dose dependent, but is ATM independent and not affected by the early G2/M checkpoint process (97). An imperfect G2/M checkpoint has been shown to contribute to chromosome instability in irradiated S and G2 phase cells [97, 98].

The article "Involvement of Nucleotide Excision and Mismatch Repair Mechanisms in Double Strand Break Repair" was published in 2009. Journal: Curr Genomics.

In the NER pathway, the evidence implicating XPC/HR23B and XPF/ERCC1 complexes in cell cycle regulation is very limited with only one report showing that XPC may be associated with the centrosomal protein centrin 2, indicating a possible linkage of XPC to cell division [99]. However, RPA and XPA proteins, which form a complex, have shown their potential roles of linking DNA damage detection and initiation of the G2/M checkpoint. *S. cerevisiae* cells with a single unrepairable DSB exhibit long, but transient arrest at G2/M. This DSB-induced arrest has been shown to be suppressed by RPA mutation, suggesting that RPA is one of the key regulators in the DNA damage-induced G2/M checkpoint [100]. In mammalian cells, RPA2, the 32kD subunit of RPA, is phosphorylated in the S and G2 phase of cell cycle through the CDC2 kinase [101] and hyperphosphorylated in cellular responses to DNA damage through ATM and DNA-PK [102], which is an essential step in chromosomal DNA repair [103]. Distinct phosphorylated forms of RPA2 have been identified in different cell-cycle stages and in response to DNA damage [102, 104]. The phosphorylated form of RPA2 in mitotic cells has been reported to exhibit less binding efficiency to double-stranded DNA and altered interaction with several DNA replication and repair proteins. *In vitro*, this type of phosphorylated RPA showed decreased binding to ATM, DNA pol alpha, and DNA-PK compared to unphosphorylated recombinant RPA [105]. In contrast, hyperphosphorylated RPA showed a high affinity for damaged duplex DNA in response to DNA damage [105]. Further studies have verified that RPA2 phosphorylated by cyclin B-CDC2 during the prometaphase of mitosis stimulates RPA2 to become hyperphosphorylated in response to mitotic DNA damage caused by bleomycin treatment, which causes single- and double-stranded breaks in DNA [106]. Mutation in RPA2 causing the lack of both CDC2 phosphorylation sites significantly suppressed the mitotic release of DNA damaged cells into G1 phase, thus decreasing cell viability [106]. These results demonstrate that RPA hyperphosphorylation regulates the cell cycle arrest induced by DNA strand breaks [106, 107].

The article "Involvement of Nucleotide Excision and Mismatch Repair Mechanisms in Double Strand Break Repair" was published in 2009. Journal: Curr Genomics.

In addition to RPA2, the depletion of RPA1, the largest subunit of RPA, results in several cell phenotypes in mammalian cells. Cells lacking RPA1 have slower S phase progression with a G2/M arrest, leading to phosphorylation of CHK2 and activation of p21 expression in human embryonic kidney and Hela cells [108, 109]. In response to camptothecin (CPT) and etoposide (ETP) induced DNA strand breaks, cells depleted of RPA1 showed a substantially accumulated number in S phase compared with G2/M arrest in wild type cells, which is consistent with the defect in DNA replication caused by RPA1 deficiency [110]. Furthermore, CPT and ETP treated RPA1-t11 Hela cells, which bear mutations at R41 and Y42, progressed into G1 phase rather than becoming arrested in G2/M phase. This suggests the critical function of the N terminal of the RPA1 containing DBD-F domain in cell cycle regulation and DNA repair [110]. This result is consistent with the defect of the G2/M checkpoint reported in *rfa1*-*t11* mutant yeast cells, which also bear a mutation in RPA [111].

The strong interaction of XPA with RPA suggests XPA as another candidate contributing to the linkage of DNA repair to cell cycle checkpoint. It has been shown that the yeast homolog of the human XPA protein, Rad14p, physically interacts with checkpoint protein Ddc1 [112]. Several studies have revealed that XPA may be involved in the cell cycle checkpoint induced by UV-generated lesions. An XPA defect abolished the phosphorylation of CHK1 and p53 in both G1 and G2 checkpoint responses to UV in primary human fibroblasts [113]. In UV irradiated cells, the modulation and phosphorylation of XPA has been showed to be ATR dependent. The XPA deficient cells with an XPA-S196 phosphorylation site mutation showed higher UV sensitivity. Moreover, cells with substituted XPA having Aspartic acid at S196 to mimic persistent phosphorylation had an increased cell survival rate compared with wild type cells after UV treatment. Therefore, the phosphorylation at S196 of XPA may be significant to the ATR-dependent checkpoint pathway in human cells [114]. Another recent report has revealed that the ATR signaling pathway is also compromised in XPA-deficient cells during S phase, as shown by defects in UV-induced phosphorylation of CHK1 and RPA using various cell lines. This lesion recognition function of XPA may be sufficient for ATR-mediated S-phase checkpoint activation since none of XPC-, CSB-, XPF- and XPG-deficient cells have impaired S-phase responses [115]. XPA has also been found to interact with a novel centrosomal protein, CEP164, at amino acids 4-97 of XPA [116]. CEP164 has been identified as a chromatin binding mediator protein that interacts with both ATR and ATM and is phosphorylated upon replication stress, UV radiation, and IR. The defect of this protein significantly reduces DNA damage-induced phosphorylation, such as phosphorylation of RPA, H2AX, MDC1, CHK2, and CHK1, and dramatically affects the G2/M checkpoint and nuclear divisions. This protein, therefore, has critical roles in both DNA damage induced checkpoint and repair [117]. Upon UV damage, XPA is required to recruit CEP164 to the damage sites. This activity was abolished by XPA mutation in XPA-deficient fibroblasts. Furthermore, XPA deficient cells showed impaired UV-induced CHK1 phosphorylation that may explain increased cell survival upon UV damage [116]. These findings provide further evidence that XPA and its interactants may mediate a critical juncture between checkpoint pathways and repair systems. Not only UV induced DNA damage, but also cisplatin induced G2/M arrest was impaired in XPA deficient fibroblast cells compared with wild type cells [118]. In our previous report, gamma irradiated XPA^KD^ cells showed increased cell cycle progression as a significantly increased percentage of bi-nucleated cells compared with irradiated control cells after cytoclasin B treatment, which arrests cells at the stage between mitosis and division [47].

The article "Involvement of Nucleotide Excision and Mismatch Repair Mechanisms in Double Strand Break Repair" was published in 2009. Journal: Curr Genomics.

In the MMR pathway, studies have shown that both MSH2 and MLH1 are involved in G2 phase cell cycle progression, suggesting that MMR-mediated cell cycle delay may be important for its function of proofreading the repaired DNA lesions prior to chromosome segregation to prevent passing critical lesions to daughter cells [119]. The MLH1 protein was reported to be involved in G2-M cell cycle checkpoint arrest induced by 5-flurouracil (5-FU) exposures, which resulted in DNA base damage and mispair lesions [120]. A recent study has demonstrated that MMR-dependent G2 arrest responses are dependent on a human MLH1/c-ABL/GADD45alpha signaling pathway [121]. The P53 pathway may be involved as well in MMR-dependent G2 arrest since it has been also shown that MLH1 has p53-response elements within the first intron and is responsive to p53 activation in normal human fibroblasts [122]. Thus, MLH1 may function beyond its MMR role as both a primary sensor to DNA damage and a critical interlink between DNA repair and cell-cycle arrest. IR treatment also generates DNA mismatches directly as well as from the DSB NHEJ repair process that is error prone [123]. Nevertheless, DSB repair involves MMR proteins, suggesting that MMR may also be the mediator in the DSB induced G2/M checkpoint. It has been demonstrated that both MLH1 and MSH2 deficient human colon carcinoma cells and murine primary embryonic fibroblasts display higher tolerance to gamma radiation induced DNA damage associated with reduced p53 dependent responses [124]. The deficient cells also exhibit a deficiency in the G2-M cell cycle checkpoint after IR exposure, as shown by fewer cells and a shorter period in G2/M arrest [124]. These findings have been further confirmed in human ovarian, endometrial and another colorectal cancer cell line with or without ectopically expressing MSH2, showing that the defect affects both X-ray and UVB induced G2 cell cycle arrest [84, 125]. Although the level of phosphorylated CDC2 (phospho-CDC2) was increased in both MMR-proficient and -deficient cell lines after IR, the amount of phospho-CDC2 rapidly decreased in MLH1 or MSH2-deficient cell lines associated with elevated progress from G2 arrest through M phase. This MMR mediated G2 cell cycle regulation may act through a decreased CDC2 phosphorylation, which upregulates CDC2 kinase activity [126] and enables cells to bypass repair lesions and being released from G2 phase. These differences in IR-induced G2 arrest between MMR-proficient and -deficient cells were found regardless of the original cell cycle stage, indicating that the regulatory effect of MMR on IR induced G2/M checkpoint arrest is dramatic [126].

## SUMMARY

In response to DNA damaging agents, complex damage response pathways are activated in mammalian cells. These pathways regulate a series of known post-insult responses: A. surveillance of DNA lesions; B. induction of cell cycle checkpoint; C. activation of DNA repair; D. maintenance of cell cycle arrest, and removal of cells with unrepaired DNA damage through apoptosis; E. proofreading and repair of minor incorrect repaired or repair intermediate lesions; and F. cellular signaling leading to either cell cycle progression or apoptosis (Fig. **1**). Although DSB repairs utilize mainly the HR and NHEJ repair machinery, a successful DSB repair process depends on precise and timely post-insult responses from A to F, and thus involves a systematically coordinated cellular network. Recent studies have confirmed that non-DSB repair mechanisms, such as NER, MMR and cell cycle regulation are highly involved in DSB repairs. These findings have revealed previously unrecognized roles for various non-DSB repair genes, in that a successful DSB repair requires both DSB repair machinery and non-DSB repair systems. The involvement of NER and MMR proteins such as RPA, XPA, MLH1 and MSH2, in both the cell cycle regulation and DSB repair, underline the importance of these proteins beyond their original pathways. These proteins regulate and maintain cell cycle arrest by either direct or indirect interaction with other cell cycle control proteins. They may also play a role in proofreading of the repaired DNA and sending signals for the repaired cells to progress through the checkpoint.

The article "Involvement of Nucleotide Excision and Mismatch Repair Mechanisms in Double Strand Break Repair" was published in 2009. Journal: Curr Genomics.

The NER and MMR proteins significantly influence the success of DSB repair through the following three steps: first, both NER and MMR physically facilitate HR/NHEJ machinery, especially in the processing of intermediates during DSB repair; second, the ability of recognizing the DNA signal strand and various small DNA structure changes may allow NER and MMR to participate in primary damage surveillance; and last but not least, several NER and MMR proteins have critical roles in signaling between primary damage reorganization, induction of cell cycle checkpoint and bridging, proofreading and permitting cell cycle progression (Fig. **1**).

Effective repair of DSBs is of great importance for the maintenance of genome stability and prevention of carcinogenesis. Incorrectly repaired lesions potentially generate mutations/recombinations that are prone to induce activation of proto-oncogenes, inactivation of tumor suppressor genes or loss of heterozygosity which can lead to carcinogenesis. Therefore, in response to DSB damage, the appropriate NER and MMR involvement is required. Failure to do so could change the outcome of post-repair scenarios: cell cycle arrest versus apoptosis; repaired, unrepaired, or misrepaired DNA; or even carcinogenesis.

## Figures and Tables

**Fig. (1).** The proposed linkage interlink between NER/MMR and DSB repair process.
